RETRACTED

# Meta-Analysis on the Anesthetic Effects of Remifentanil plus Dexmedetomidine versus Remifentanil Alone in Cardiac Surgery

**DOI:** 10.1155/2022/1077980

**Published:** 2022-09-28

**Authors:** Xiao-Lin Zeng, Jun-Hua Liao, Hui-Sheng Zhong, Xin-Hua Yin, Rui Wang, Jiu-Ping Liang, Zheng-Sheng Zhang

**Affiliations:** ^1^Department of Cardiology, Shenzhen University General Hospital, Shenzhen, China; ^2^Guangzhou Yujia Biotechnology Co., Ltd., Guangzhou, China; ^3^Cardiac Surgery Center, The First Affiliated Hospital of Gannan Medical University, Jiangxi, China; ^4^Department of Radiology, Shenzhen Bao'an District Songgang People's Hospital, Shenzhen, China; ^5^Department of Cardiology, Pingshan District People's Hospital of Shenzhen, Pingshan General Hospital of Southern Medical University, Shenzhen, Guangdong, China

## Abstract

In this study, we performed a meta-analysis to investigate the anesthesia effects of remifentanil plus dexmedetomidine versus remifentanil alone in cardiac surgery. Literature search was performed on PubMed, Web of Science, Embase, China Knowledge Infrastructure, Wanfang Data, and other databases for relevant literature published in English or Chinese before October 2021. A total of 17 studies, consisting of 1350 patients, were included in this study. Of these, 10 studies showed that remifentanil plus dexmedetomidine had a good anesthesia effect in cardiac surgery (OR = 3.61, 95% CI: 1.73, 7.52, *P* < 0.001), and 8 studies showed that the Ramsay score test of anesthesia (SMD = 0.88; 95% CI: -0.77, 2.53; *P* < 0.001) in the experimental group was better than that in the control group. In addition, changes in the hemodynamic heart rate (SMD = −0.74; 95% CI: -1.41, -0.07; *P* < 0.001) and mean arterial pressure (SMD = −0.18; 95% CI: -0.72, 0.36; *P* < 0.001) of the two groups of anesthesia were counted in 17 studies, which also showed that the anesthesia effect of remifentanil plus dexmedetomidine was good. Thus, remifentanil plus dexmedetomidine may be a more promising option for cardiac surgery anesthesia than remifentanil alone.

## 1. Introduction

In recent years, the prevalence rate of cardiac diseases in China has continued to rise, and the current number of cardiovascular diseases has reached about 290 million [1], indicating that an increasing number of patients are requiring cardiac surgery. According to statistics, the number of cardiac surgery has increased from 90,812 cases in 2004 to 207,881 cases in 2013, with an annual growth rate of 9.64% [2]. However, cardiac surgery is very complicated and difficult to perform. Therefore, one of the goals of the induction phase of general anesthesia in cardiac surgery is to inhibit intubation stress response; keep control of mean arterial pressure (MAP), heart rate (HR), and other hemodynamic indexes relatively stable in the normal range; and improve anesthesia and analgesic effects [3].

RETRACTED

Remifentanil is an ultrashort-acting *μ*-opioid receptor agonist widely used in cardiac surgery anesthesia due to its rapid onset, short half-life, and metabolism independent of liver and kidney function [4]. However, some studies have found that the use of remifentanil for anesthesia for long durations in surgery could continuously reduce the MAP and HR of patients, followed by large fluctuations in hemodynamics. In addition, it can also increase the sensitivity of patients to pain and reduce tolerance to surgery, significantly reducing the anesthetic and muscle relaxation effects and increasing the incidence of adverse reactions [5]. In comparison, dexmedetomidine, a highly selective *α*2AR agonist, has been widely used as an adjuvant drug for clinical anesthesia in China and abroad [6]. It can stimulate *α*2 adrenergic receptors in the central and peripheral nervous systems, tissues, and organs and effectively inhibit the conduction of excitation signals in the vagus nerve, thereby stabilizing blood pressure and HR. It was also shown to possess sedative, analgesic, and hypnotic functions, as well as inhibition of sympathetic nerve activity [7], without causing respiratory depression. Additionally, dexmedetomidine was reported to reduce patients' nerve sensitivity to pain, inhibit the occurrence of stress response, and thus improve the anesthetic effect [8]. Although numerous studies have shown that remifentanil combined with dexmedetomidine positively affects anesthesia in cardiac surgery [9–11], its anesthetic and hemodynamic effects still need to be systematically and comprehensively evaluated.

We hypothesized that remifentanil combined with dexmedetomidine would potentially be conducive to preventing the cardiovascular system's adverse reactions compared with remifentanil alone. Thus, we systematically analyzed current literature to evaluate the anesthetic effects, Ramsay score, MAP, and HR as evaluation indexes to determine the anesthetic effects of remifentanil combined with dexmedetomidine and remifentanil alone in cardiac surgery.

## 2. Materials and Methods

### 2.1. Literature Retrieval

Databases such as PubMed, Web of Science, and Embase were used for literature search using search words “remifentanil combined with dexmedetomidine” and “(remifentanil) and (dexmedetomidine) and (cardiac surgery)” in English. Also, Chinese databases such as the China Knowledge Network and Wanfang Data databases were searched using the search terms “remifentanil combined with dexmedetomidine,” “cardiac surgery,” and “anesthesia” in Chinese. A thorough search of relevant literature from the references of eligible studies was also performed. For this study, the conference and abstract articles of some literature were also selected.

RETRACTED

### 2.2. Inclusion and Exclusion Criteria

The study inclusion criteria were based on participants, interventions, comparison, outcomes, and study (PICOS) design programs and were as follows: (1) *participants (P)*: patients undergoing cardiac surgery based on a definite diagnosis; (2) *interventions and comparisons (I, C)*: experimental group: patients undergoing cardiac surgery were anesthetized with remifentanil combined with dexmedetomidine; control group: patients undergoing cardiac surgery were anesthetized with remifentanil; (3) *outcomes (O)*: the excellent and good rate of anesthesia [12] (excellent: no response to stimuli, deep sleep; good: agile response to stimuli, arousable to obey instructions, light sleep; poor: irritability without pressing, anxiety), Ramsay score, HR, and MAP, etc.; and (4) *study designs (S)*: all studies compared the anesthetic effects of remifentanil combined with dexmedetomidine or remifentanil alone in patients undergoing cardiac surgery. The study exclusion criteria were (1) irrelevant articles, (2) review articles, (3) duplicate studies, and (4) incomplete data, defective design, and unclear study conclusions.

### 2.3. Literature Quality Evaluation and Data Extraction

The risk of bias in each identified study was assessed using the Cochrane Collaboration's tool [13], which considered six different domains: (1) random sequence generation (selection bias), (2) allocation concealment (selection bias), (3) blinding of participants and personnel (performance bias), (4) blinding of outcome assessment (detection bias), (5) incomplete outcome data (attrition bias), and (6) selective reporting (reporting bias). Two researchers independently performed literature evaluation and data extraction, and disagreements were resolved by discussion and consultation with a third researcher.

### 2.4. Statistical Analysis

The Stata 16.0 was used for statistical analysis. Cochrane's *Q* test and *I*^2^ statistics were used to evaluate the heterogeneity of the included studies. If *P* < 0.05 and *I*^2^ > 50%, the random effects model was selected for the meta-analysis; otherwise, the fixed effects model was used. In addition, the results of categorical variables were reported as odds ratio (OR) and 95% confidence interval (CI), while the results of numerical variables were reported as standardized mean difference (SMD) and 95% CI. *P* < 0.05 indicated that the difference was statistically significant. Moreover, sensitivity analysis was used to evaluate the reliability of the meta-analysis results, and the funnel plot was used to analyze the possibility of publication bias.

RETRACTED

## 3. Results

### 3.1. General Information of Included Studies

A total of 818 articles were initially retrieved, of which 151 were selected after excluding unqualified papers by evaluating their titles, abstracts, and full texts. In a later review of the bias of some studies and the requirements of research methods, only 17 studies [12, 14–29] met the selection criteria, including 2 foreign literature and 15 Chinese literature. A total of 1350 patients were divided into the remifentanil combined with dexmedetomidine group, and 675 were in the control group. The characteristics of the included literature are shown in Figure 1 and Table 1.

### 3.2. Analysis Results

#### 3.2.1. Excellent and Good Rate of Anesthesia

The outcome variable of the 10 studies [12, 15–17, 19, 22, 23, 25, 26, 29] included was reported as excellent and good rate of anesthesia. The data after merging showed that the heterogeneity of each study was small (*I*^2^ = 68.9%, *P* = 0.001). Therefore, the random effects models were adopted. The results showed that the excellent and good rate of anesthesia in the experimental group was higher than that in the control group, and the difference was statistically significant (OR = 3.61, 95% CI [1.73, 7.52], *P* = 0.001) (Figure 2(a)).

#### 3.2.2. Ramsay Score of Anesthesia

Eight studies [15, 16, 18, 19, 21, 22, 26, 29] reported on the Ramsay score of anesthesia, with the results of each study showing significant heterogeneity (*I*^2^ = 98.8%, *P* < 0.001). The random effects models were also used for analysis. According to the meta-analysis, the Ramsay score of anesthesia in the experimental group was significantly lower than that in the control group (SMD = 0.88, 95% CI [−0.77, 2.53], *P* < 0.001) (Figure 2(b)).

#### 3.2.3. Hemodynamic Indexes of Anesthesia

All the 17 included studies [12, 14–29] recorded the patients' hemodynamic HR during anesthesia in both groups. The obtained heterogeneity test result was *I*^2^ = 96.9% (*P* < 0.001). By adopting the random effects models, the results showed no statistical differences in the hemodynamic HR during anesthesia between the two groups (SMD = −0.74, 95% CI [-1.41, -0.07], *P* < 0.001) (Figure 3(a)).

In addition, the 17 studies [12, 14–29] recorded the changes in MAP during anesthesia in the two groups, and the heterogeneity test result was *I*^2^ = 95.6% (*P* < 0.001). Random effects models were applied, and the meta-analysis indicated no statistically significant differences in the results (SMD = −0.18, 95% CI [-0.72, 0.36], *P* < 0.001). We also observed that the hemodynamics of remifentanil combined with dexmedetomidine in the test group was more stable than that in the control group, thus indicating improved safety of anesthesia when using remifentanil plus dexmedetomidine (Figure 3(b)).

RETRACTED

#### 3.2.4. Sensitivity Analysis

The sensitivity analysis results showed that after changing the inclusion criteria, excluding low-quality studies, and removing the maximum and minimum weights, the merged results showed little changes from the original merged results, indicating a low sensitivity and that the results of the meta-analysis were reliable. Sensitivity analysis is shown in Figures 4(a) and 4(b) and Figures 5(a) and 5(b).

#### 3.2.5. Publication Bias

The funnel plot was used to detect possible publication bias. The funnel diagram, including SMD of MAP and HR, showed that the scattered points were basically symmetrical about the axis of symmetry, thus indicating no significant publication bias in all studies (Figures 6(a) and 6(b)).

## 4. Discussion

Although previous studies demonstrated that remifentanil combined with dexmedetomidine was safe and effective for anesthesia in cardiac surgery, the hemodynamic effects of this combined regimen remained to be systematically and comprehensively evaluated. In this meta-analysis of 17 studies, the included literature had similar research methods and were retrospective studies, with little heterogeneity in outcome evaluation indicators and high comparability. Among them, 10 studies evaluated the excellent and good rate of anesthesia. The results showed excellent and good anesthesia rates between 90.90% and 96.00%, respectively, in the test group and 48.00% and 69.69%, respectively, in the control group. According to the meta-analysis, remifentanil combined with dexmedetomidine had an excellent and good anesthesia rate and significantly better anesthetic effects than remifentanil alone.

We believe that the superior anesthetic effects of the combination regimen compared with the single drug might be related to dexmedetomidine being able to reduce the sensitivity of patients' nerves to remifentanil-induced pain, and at the same time, it played an important role in controlling the occurrence of stress response and improving anesthetic effects [8]. The results of the included studies [12, 14, 18, 20–22, 24] also showed that the time of anesthetic maintenance and tracheal extubation in the test group was significantly longer than that in the control group, and the anesthetic onset time was significantly shorter than in the control group, which were significantly different for the two groups. It was further proven that the experimental group could improve the effectiveness of surgical anesthesia.

RETRACTED

Eight studies reported on the Ramsay scores of anesthesia, showing lower Ramsay scores in the test group than in the control group. The meta-analysis showed that remifentanil combined with dexmedetomidine could significantly reduce the Ramsay score of anesthesia than remifentanil alone. Regarding the reasons for the decrease in the Ramsay score, some relevant studies have found that dexmedetomidine could activate *α*2 adrenergic receptors in the central and peripheral nervous systems as well as tissues and organs, exerting positive effects on sedation and analgesia [30]. Others have proposed that the improved analgesic effects provided by dexmedetomidine might be due to modulation of catecholamine release, reduction of catecholamine concentrations during the perioperative period and synergistic analgesic effects of opioids, and weakness of stress response to surgery and anesthesia [31].

The 17 studies included reported the MAP and HR in the hemodynamics of anesthesia in the two groups. Under the condition that there were no significant differences in the MAP and HR between the two groups before surgery, however, they both changed to different extents during surgery. The fluctuation range of MAP and HR in the test group was less than that in the control group; that is, their overall trend in the test group was more stable, indicating that remifentanil combined with dexmedetomidine could improve the stability of hemodynamics, HR, and MAP of patients, and could be conducive to prevent the cardiovascular system from adverse reactions caused by severe fluctuation of blood pressure and HR during surgery. We believe that these effects were associated with the ability of dexmedetomidine to activate the *α*2 receptor in the locus coeruleus of the central nervous system and antagonize sympathetic stimulations to maintain hemodynamic stability during surgery [30]. Besides, other researchers have reported that dexmedetomidine helps keep hemodynamic stability in children undergoing cardiac surgery [32]. Previous studies [12, 21, 23, 28] also found that dexmedetomidine could significantly reduce the remifentanil dosage by about 17.29%. Moreover, some studies have confirmed a reduction in opioid use when comparing dexmedetomidine for sedation with prednisone or benzodiazepines [33], suggesting that dexmedetomidine could lessen the adverse effects caused by excessive anesthetic use. Nonetheless, like some other opioids, the side effects of remifentanil include respiratory depression, bradycardia, decreased blood pressure, muscle rigidity, seizures, nausea, and vomiting, which are all dose-related. Consequently, appropriate dosages of anesthetic induction drugs might be selected based on individual differences to guard against the side effects of inappropriate remifentanil doses. Dexmedetomidine also has side effects, such as hypotension and bradycardia, with an increased incidence of approximately 3.4 times compared with events without dexmedetomidine, suggesting that HRs should be carefully monitored when dexmedetomidine is used during anesthesia of cardiac surgery [34].

RETRACTED

This meta-analysis had certain limitations that should be described. First, the sample size of the included studies and the overall population range of the sample were relatively small, and most of the included studies were from China. Thus, there may be certain bias and low test efficiency, and the study conclusions could not be extrapolated to all populations. Second, no blind or allocation concealment methods were used in the study to control information bias, which might have had certain effects on the internal authenticity of the results. Lastly, there are many anesthesia methods for cardiac surgery in clinical practice, but in this study, only remifentanil was used as the control group, which could not represent other clinical anesthesia schemes, such as sufentanil combined with propofol. Still, the comparison of remifentanil combined with dexmedetomidine with other anesthesia schemes was lacking, which affected the extrapolation of the results in clinical application.

## 5. Conclusion

In summary, remifentanil combined with dexmedetomidine for cardiac surgery was shown to improve the excellent and good rate of anesthesia, reduce the Ramsay score of anesthesia, decrease severe changes in HR and MAP, and enhance the stability of hemodynamics, thereby achieving significantly better anesthetic effects compared with remifentanil only. In addition, the combined regimen not only prolonged the duration of anesthesia and the time of tracheal extubation but also shortened the onset time of anesthetics. Meanwhile, dexmedetomidine was shown to lower the dosage of remifentanil, thus reducing potential adverse effects related to excessive anesthetic use.

## Figures and Tables

**Figure 1:** Flowchart of the study selection process for identifying eligible studies.

**Figure 2:** Forest plot showing the (a) excellent and good rate score of anesthesia and (b) Ramsay score of the two groups.

**Figure 3:** Forest plot of the (a) mean arterial pressure and (b) heart rate of the two groups.

**Figure 4:** Sensitivity analysis of the (a) excellent and good rate score of anesthesia rate and (b) Ramsay score of anesthesia.

RETRACTED

**Figure 5:** Sensitivity analysis of (a) mean arterial pressure and (b) heart rate of the two groups.

**Figure 6:** Funnel plot of the (a) mean arterial pressure and (b) heart rate of the two groups.

**Table 1:** The basic characteristics of the included literature.

No.	First author	Year	Country	Sample time (year.month)	No. patients treat/con	Age (mean ± SD)		Sex ratio (male/female)		Study design	Outcome measured
						Treatment group	Control group	Treatment group	Control group		
1	Lei Jiaxiu [14]	2018	China	2017.3~2017.9	75/75	43.92 ± 11.28	43.58 ± 11.73	43/32	41/34	Retrospective	①+②
2	Huo Chengjuan [15]	2019	China	2017.6~2018.8	60/60	46.56 ± 2.48	46.53 ± 2.42	37/23	36/24	Retrospective	① + ② + ③
3	Hao Meiling [12]	2017	China	2014.1~2015.12	30/30	46.0 ± 2.0	45.5 ± 2.1	17/13	19/11	Retrospective	① + ②
4	Ma Yong [16]	2016	China	2012~2015	50/50	35 ± 1.4	36 ± 1.1	30/20	28/22	Retrospective	① + ② + ③
5	Liang Yan [17]	2018	China	2015.10~2017.10	33/33	38.74 ± 2.39	38.56 ± 2.21	19/14	20/13	Retrospective	① + ②
6	Zhong Baolin [18]	2015	China	2013.4~2015.1	50/50	44.13 ± 7.13	44.01 ± 7.24	28/22	26/24	Retrospective	① + ② + ③
7	Jing Guangxia [19]	2014	China	2012.1~2014.1	60/60	49.60 ± 1.82	47.70 ± 1.77	33/27	33/27	Retrospective	① + ② + ③
8	Zhao Jun [20]	2020	China	2017.5~2018.7	31/31	49.52 ± 2.48	49.56 ± 2.51	18/13	17/14	Retrospective	① + ②
9	Yang Bing [21]	2018	China	2015.10~2017.10	40/40	44.65 ± 7.11	44.71 ± 7.09	23/17	22/18	Retrospective	① + ② + ③
10	Wang Daofu [22]	2016	China	2013.12~2015.9	50/50	44.08 ± 7.21	44.63 ± 7.12	29/21	28/22	Retrospective	① + ② + ③
11	Jia Yanjie [23]	2018	China	2016.5~2017.2	33/33	38.56 ± 7.48	38.41 ± 7.34	18/15	19/14	Retrospective	① + ②
12	Wang Xiaoying [24]	2018	China	2015.10~2018.10	20/20	59.74 ± 5.19	59.79 ± 5.16	11/9	10/10	Retrospective	① + ②
13	Wang Li [25]	2018	China	2016.10~2018.2	30/30	45.53 ± 8.92	45.06 ± 9.01	18/12	19/11	Retrospective	① + ②
14	He Xiaoxia [26]	2019	China	2018.1~2018.12	35/35	49.13 ± 4.52	48.42 ± 4.96	18/17	20/15	Retrospective	① + ② + ③
15	Zhi Wang [27]	2017	China	2015.1~2015.12	48/48	56.43 ± 6.57	56.38 ± 6.47	25/23	26/22	Retrospective	① + ②
16	Mediha Türktan [28]	2017	Turkey.	2014.12~2015.8	30/30	59.83 ± 14.22	53.90 ± 15.43	17/13	21/9	Retrospective	① + ②
17	Jin Sun Cho [29]	2014	Korea.	NR	45/45	55.2 ± 8.7	56.3 ± 9.3	36/9	36/9	Retrospective	① + ② + ③

Note: ①: mean arterial pressure, MAP; ②: heart rate, HR; ③: Ramsay score; Treat: treatment; Con: control; NR: not reported.

## Data Availability

The data used to support the findings of this study are available from the corresponding authors upon request.

## Abbreviations

CI: Confidence interval
HR: Heart rate
I, C: Interventions and comparisons
MAP: Mean arterial pressure
O: Outcomes
OR: Odds ratio
P: Participants
S: Study designs
SMD: Standardized mean difference.
